# The Anion Gap and Mortality in Critically Ill Patients with Hip Fractures

**DOI:** 10.1155/2022/1591507

**Published:** 2022-07-06

**Authors:** Xiao-Bo Zhang, Wu-Bin Shu, A-Bing Li, Guan-Hua Lan

**Affiliations:** Department of Orthopedics, Ningbo Yinzhou No. 2 Hospital, Ningbo 315100, Zhejiang, China

## Abstract

**Objectives:**

Epidemiological evidence suggests that anion gap (AG) has been reported to serve as an independent predictor for mortality in different diseases. We studied the effect of AG on both short and long-term mortalities in critically ill patients with hip fracture.

**Methods:**

A large clinical database was utilized to perform retrospective cohort analysis. AG was subdivided into three groups. The Cox proportional hazards regression model was employed to approximate the hazard ratio (HR) with a confidence interval (CI) of 95% for the link between AG and mortality. 30-day mortality is the primary outcome, while 90-day and 1-year mortalities represented our secondary outcomes for this study.

**Results:**

The participants in this study were that who provided essential data on AG and the number of patients with hip fractures was 395, and they were all aged ≥16 years. The participants comprised 199 (50.4%) females as well as 196 (49.6%) males with an average age of 71.9 ± 19.4 years, and a mean AG of 12.4 ± 3.3 gmEq/L. According to an unadjusted model for 30-day all-cause mortality, the HR (95% CI) of AG ≥ 12.5 gmEq/L was 1.82 (1.11, 2.99), correspondingly, compared to the reference group (AG < 12.5 gmEq/L). This correlation was still remarkable after adjustment for *r* age, sex, race, SBP, DBP, WBC, heart failure, and serum chloride (HR = 1.70, 95% CI: 1.02–2.02; 2.82). For 90-day all-cause mortality, a similar correlation was observed.

**Conclusions:**

We noted that AG was an independent indicator of both short and long-term mortalities among hip fractures individuals in this retrospective single-center cohort study. AG is a simple, readily available, and inexpensive laboratory variable that can serve as a possible risk stratification tool for hip fracture.

## 1. Introduction

Hip fractures pose a worldwide health burden, and it is not only frequently encountered in the acute orthopedic departments but also correlated to morbidity and mortality [1, 2]. These patients tend to have an increased risk of developing postoperative complications, disability, and high 1-year mortality estimated at 30% [3]. Improvements in life expectancies all over the world lead to the fact that around 1.5 million hip fractures will occur each year [3]. By the end of 2025, 6.3 million individuals will suffer from hip fractures worldwide, posing a huge burden on their caregivers and society, respectively, ranking hip fractures among the major causes of morbidity globally. These fractures have been linked to short and long-term mortalities. The current approximates of mortality during the first postoperative month fall within 5–10%, while the first year can reach up to 36%. Based on these reservations, it is imperative to discover early prognosis and preventive strategies to address the problem of high-risk hip fractures.

The serum anion gap (AG) arises when there is an excessive synthesis of organic acid anions and/or an equivalent reduction in anion secretion [4, 5]. AG is a potential parameter that can be computed mathematically and utilized in diagnosing different metabolic acidosis [6, 7]. The numerous studies conducted recently have revealed that anion gap (AG) has a promising predictive value for various ailments, for instance, heart failure [8], coronary heart disease [9], and myocardial infarction [10, 11]. We carried out this research to ascertain the link between AG and mortalities related to hip fractures and to verify whether AG is a predictive factor for the prognosis among hip fracture-ICU patients, utilizing patient data from Medical Information Mart for Intensive Care III (MIMIC-III) [12]. We anticipated that a simple AG might be the first laboratory predictor of prognosis in individuals with hip fractures and that it could be employed as a supplementary tool to detect individuals with hip fractures who are at high risk of poor prognosis.

## 2. Methods

### 2.1. Study Population

The experiment followed the Strengthening the Reporting of Observational Studies in Epidemiology (STROBE) statements [13, 14]. Data were obtained from MIMIC-III version 1.4 [15], which was utilized to record the following variables: vital signs, demographic data, medications, and other vital items of 53,423 different hospital admissions to ICU in the Beth Israel Deaconess Medical Center (BIDMC) in Boston ranging from 2001 to 2012. The application for data use has been approved by the Massachusetts Institute of Technology (MIT) as well as the Institutional Review Boards. Researchers passed the online course “Data or Specimens Only Research.”

Patients with hip fractures (ICD-9-CM (International Classification of Disease, 9th revision, clinical modification)) more than 16 years old at the time of admission and hospitalized for more than 1 day were retrieved from the MIMIC-III database. Patients were eliminated if they spent less than 48 hours in the ICU and had no data on AG during the initial 24 hours of admission.

### 2.2. Variable Extraction

In order to screen every patient, the researcher utilized Structured Query Language with PostgreSQL. We obtained the patient's demographic data (age, patient gender, and race), laboratory characteristics, vital signs, comorbidities, and scoring systems. Within 24 h after patients' admission to ICU, the vital signs were obtained, including SPO_2_, systolic blood pressure (SBP), heart rate, and diastolic blood pressure (DBP). Hemoglobin, white blood cell (WBC) count, hematocrit, serum potassium, serum glucose, and serum chloride over the first 24 hours were the laboratory measurements.

### 2.3. Outcome

The 30-day mortality served as our primary outcome, while the 90-day mortality represented secondary outcomes. The date when patients were admitted was the initial date for commencing follow-up, and all subjects were studied for 90-day. The patient's first date of admission to a hospital facility until the date of death was the observation time. The Social Security Death Index records provided accurate dates for death.

### 2.4. Statistical Analysis

To investigate the link between AG and the outcome of patients with hip fractures, the process of statistical analysis is split into four steps. First, the subjects were further subdivided into 2 groups on the basis of AG. The continuous data were presented as the mean ± standard deviation (SD), while categorical variables were presented as either frequency or percentage. Differences in baseline characteristics between tertiles of AG were examined using the Kruskal–Wallis H test in continuous variables and *χ*^2^ test for categorical variables. Second, the COX regression was established to evaluate the correlation between AG and the outcome of patients with hip fractures. There were no covariates adjustments in model A, while in model B, only sex, age, and race required adjustments and model C adjusted confounders age, sex, race, SBP, DBP, WBC, heart failure, and serum chloride. Third, we performed smooth curve fitting using a penalized spline approach to detect the nonlinearity of AG and the outcome of patients with hip fractures. R software (version 3.6.1, http://www.r-project.org) was used for all of the investigations. All *p* values were two-sided, and *P* values <0.05 were statistically significant.

## 3. Result

### 3.1. Baseline Characteristics of Selected Participants

The participants in this study were that who provided essential data on AG and the number of patients with hip fractures was 395, and they were all aged ≥16 years. The participants comprised 199 (50.4%) females and 196 (49.6%) males with an average age of 71.9 ± 19.4 years and a mean AG of 12.4 ± 3.3 gmEq/L.

Table 1 provides the summary of sample characteristics in relation to the 30-day mortality of our sample. The patients in the 30-day mortality group were older and had significantly higher APSIII score, BUN, hematocrit, creatinine, and AG as compared to those in the survival group. Vital signs, including DBP, and temperature were lower in the mortality group. We analyzed the baseline characteristics of the patients according to AG as given in Table 2. The data showed that patients with higher AG were older, had higher APSIII scores, 30-day mortality, and 90-day mortality and higher rate of hypertension, compared to those with the lower AG group. Moreover, the patients had higher WBC, platelet, hemoglobin, hematocrit, creatinine, and BUN.

### 3.2. Association between AG and Outcome

We performed smooth curve fitting and evaluated linear relationships between AG and 30-day mortality for patients with hip fractures to illustrate linearity of AG and 30-day mortality (Figure 1).

In our research, we developed various models to evaluate the independent impacts of AG and the hip fractures subjects' outcomes after controlling for other possible confounders.  Table 3 provides effect sizes (HR) and 95% CIs. According to an unadjusted model for 30-day all-cause mortality, the HR (95% CIs) of the AG°≥°12.5°gmEq/L was 1.82 (1.11, 2.99), correspondingly, compared to the reference group (AG°<°12.5°gmEq/L). This correlation was still remarkable after adjustment for *r* age, sex, race, SBP, DBP, WBC, heart failure, and serum chloride (HR = 1.70, 95% CI: 1.02–2.02; 2.82). On the other hand, for 90-day all-cause mortalities, a similar correlation was observed.

## 4. Discussion

Hip fractures are prevalent traumas especially among geriatric patients upon admission to the hospital facility and in surgical care [16]. As the population becomes older, the statistics of geriatrics diagnosed and undergoing femur fracture surgeries is sharply increasing. Femur fractures are related to a mortality rate of 6.2%–8.3% within the first 30 days postoperative and 30% mortality during one year [17, 18].

AG is a parameter that can be mathematically derived, and it serves as the simplest approach for evaluating patients on the basis of their acid-base status [19], which is calibrated as the difference between serum cation and anion concentration measurements [20, 21]. The AG is among the frequently and widely utilized biomarkers, and it is regularly investigated for all intensive care unit patients upon admission [22]. AG of critically sick individuals is thought to be a sensitive and specific technique for determining prognosis and mortality risk. A preceding research has suggested that an elevation in AG might be associated with a better patient prognosis in a variety of disorders [11, 23, 24]. After correcting for pertinent confounding variables, AG was revealed to be a remarkable predictor of poor outcomes among patients with hip fractures in this investigation.

Moreover, preoperative acidosis can be linked to coagulopathy [8]. It is depicted that acidosis is a potential cause of coagulopathy, and hemorrhage resulting from coagulopathy increases intraoperative mortality among patients with ruptured hip fractures [25]. Various levels of AG are substantially related to different incidence rates of coagulopathy, which could provide supportive evidence for this hypothesis. Additionally, acid-base disruption, it is affirmed that among geriatrics, the increased AG level is a mortality prognostic factor, since it is linked to hypertension, decreased renal function, and low cardiorespiratory fitness. These factors may have a detrimental impact on hip fracture patients' prognoses and lead to higher AG and thus higher mortality.

The MIMIC-III is a publicly accessible database developed to offer huge amounts of digital health information accessibility freely. After accomplishing the requisite training course, researchers are allowed to utilize MIMIC-III in their clinical studies. As a result, researchers will be able to utilize sophisticated electronic health records to determine clinical outcomes and confirm published findings in ICU settings.

Our research has a few drawbacks. First, as this was a retrospective study, it is likely to be prone to selection bias. Second, the diagnosis was made using the ICD-9 code for hip fractures, which might contribute to bias. Third, we retrieved AG data for individuals based on the test performed upon their hospitalization to the ICU and did not evaluate patterns in AG changes, which may have influenced the results' reliability. Finally, because this was an observational study, we were unable to validate the possible mechanism linking a greater AG to hip fracture severity and prognosis.

## 5. Conclusion

We discovered that AG was an independent predictor of both short and long-term mortalities among hip fracture patients in this retrospective single-center sample. The AG, a simple, easily available, and affordable laboratory variable, may have merit for risk categorization of hip fractures.

## Figures and Tables

**Figure 1:** The relationship between AG and 30-day mortality for patients with hip fractures.

**Table 1:** Baseline characteristics of the study population.

Characteristics	Survival	Mortality	*P* value
*N*	331	64	

Age, years	69.6 ± 20.0	83.8 ± 10.0	<0.001

Sex, *n* (%)			0.008
Male	157 (47.4%)	42 (65.6%)	
Female	174 (52.6%)	22 (34.4%)	

Ethnicity, *n* (%)			0.032
White	258 (77.9%)	59 (92.2%)	
Black	16 (4.8%)	1 (1.6%)	
Others	57 (17.2%)	4 (6.2%)	

Vital signs			
SBP (mmHg)	118.3 ± 15.6	116.2 ± 20.8	0.135
DBP (mmHg)	58.1 ± 10.6	54.2 ± 12.7	0.009
MAP (mmHg)	75.4 ± 10.8	73.2 ± 12.8	0.115
Heart rate (bpm)	88.7 ± 15.6	87.0 ± 18.0	0.403
Respiratory rate (t/min)	18.5 ± 3.6	20.7 ± 4.4	0.403
Temperature (°C)	36.9 ± 0.6	36.6 ± 0.9	0.027
SpO_2_ (%)	97.1 ± 3.6	96.6 ± 2.7	0.053

Comorbidities			
Heart failure, *n* (%)	92 (27.8%)	38 (59.4%)	<0.001
Hypertension, *n* (%)	48 (14.5%)	12 (18.8%)	0.375
Obesity, *n* (%)	13 (3.9%)	5 (7.8%)	0.169
Infection, *n* (%)	151 (45.6%)	36 (56.2%)	0.109

Laboratory parameters			
AG	12.3 ± 3.2	13.3 ± 3.5	<0.001
WBC, 10^9^/L	10.2 ± 6.1	11.4 ± 5.8	0.079
Platelet, 10^9^/L	185.2 ± 101.4	203.1 ± 118.6	0.524
Hemoglobin (g/dl)	9.3 ± 1.8	9.7 ± 1.8	0.094
Hematocrit (%)	27.0 ± 5.4	28.8 ± 5.5	0.005
Creatinine (mg/dl)	1.2 ± 1.1	1.2 ± 0.8	0.013
BUN (mg/dl)	23.1 ± 15.6	31.0 ± 17.8	<0.001
Lactate (mol/L)	1.8 ± 1.1	2.2 ± 1.6	0.524

Scoring systems			
APSIII score	45.7 ± 17.9	59.5 ± 22.2	<0.001
Length of stay in ICU	4.0 ± 5.2	4.1 ± 4.3	0.626

AG, anion gap; SBP, systolic blood pressure; DBP, diastolic blood pressure; MAP, mean arterial pressure; ICU, intensive care unit; WBC, white blood cell; BUN, blood urea nitrogen.

**Table 2:** Baseline characteristics of the study population according to AG.

	AG		*P* value
	<12.5	≧12.5	
*N*	225	170	

Age, years	69.5 ± 21.3	75.1 ± 16.0	0.026

Sex, *n* (%)			0.459
Male	117 (52.0%)	82 (48.2%)	
Female	108 (48.0%)	88 (51.8%)	

Ethnicity, *n* (%)			0.088
White	189 (84.0%)	128 (75.3%)	
Black	7 (3.1%)	10 (5.9%)	
Others	29 (12.9%)	32 (18.8%)	

Vital signs			
SBP (mmHg)	118.2 ± 16.8	117.9 ± 16.1	0.874
DBP (mmHg)	57.3 ± 10.4	57.6 ± 11.9	0.723
MAP (mmHg)	75.1 ± 11.2	74.9 ± 11.1	0.773
Heart rate (bpm)	89.5 ± 16.0	86.9 ± 16.0	0.129
Respiratory rate (t/min)	18.7 ± 3.9	19.2 ± 3.8	0.403
Temperature (°C)	36.9 ± 0.6	36.7 ± 0.7	0.013
SpO_2_ (%)	97.5 ± 2.0	96.4 ± 4.8	<0.001

Comorbidities			
Heart failure, *n* (%)	66 (29.3%)	64 (37.6%)	0.082
Hypertension, *n* (%)	22 (9.8%)	38 (22.4%)	<0.001
Obesity, *n* (%)	9 (4.0%)	9 (5.3%)	0.541
Infection, *n* (%)	104 (46.2%)	83 (48.8%)	0.608

Laboratory parameters			
WBC, 10^9^/L	9.6 ± 4.5	11.4 ± 7.4	0.010
Platelet, 10^9^/L	178.5 ± 90.5	200.7 ± 119.7	0.069
Hemoglobin (g/dl)	9.1 ± 1.6	9.6 ± 2.0	<0.001
Hematocrit (%)	26.4 ± 5.0	28.4 ± 6.0	<0.001
Creatinine (mg/dl)	0.9 ± 0.4	1.6 ± 1.5	<0.001
BUN (mg/dl)	20.0 ± 11.7	30.3 ± 19.2	<0.001
Lactate (mol/L)	1.7 ± 0.8	2.1 ± 1.5	0.021

Scoring systems			
APSIII score	44.7 ± 17.2	52.3 ± 21.1	<0.001
Length of stay in ICU	4.0 ± 5.2	4.1 ± 4.3	0.626
30-day mortality	28 (12.4%)	36 (21.2%)	0.020
90-day mortality	42 (18.7%)	48 (28.2%)	0.025

AG, anion gap; SBP, systolic blood pressure; DBP, diastolic blood pressure; MAP, mean arterial pressure; ICU, intensive care unit; WBC, white blood cell; BUN, blood urea nitrogen.

**Table 3:** HR (95% CIs) for all-cause mortality across groups of AG.

	Model A		Model B		Model C	
	HR (95% CIs)	*P* value	HR (95% CIs)	*P* value	HR (95% CIs)	*P* value
30-day all-cause mortality						
<12.5	1.0		1.0		1.0	
≥12.5	1.82 (1.11, 2.99)	0.0170	1.71 (1.04, 2.82)	0.0335	1.70 (1.02, 2.82)	0.0433

90-day all-cause mortality						
<12.5	1.0		1.0		1.0	
≥12.5	1.63 (1.08, 2.47)	0.0201	1.49 (1.05, 2.26)	0.0391	1.50 (1.01, 2.34)	0.0458

Model A covariates were adjusted for nothing; model B covariates were adjusted for age, sex and race; model c covariates were adjusted for age, sex, race, SBP, DBP, WBC, heart failure, serum chloride.

## Data Availability

The data used to support this study are available from the corresponding author upon request.
